This article has been retracted.

# Identification of Differentially Expressed Long Noncoding RNAs as Functional Biomarkers and Construction of Function Enrichment Network in Oral Squamous Cell Carcinoma

**DOI:** 10.1155/2022/1572249

**Published:** 2022-06-25

**Authors:** Fang Xiao, Ke Wang, Yaojun Chen, Yanzhen Zhang

**Affiliations:** ^1^Department of Dentistry, Hangzhou Linping First People's Hospital, Hangzhou, Zhejiang 311100, China; ^2^Department of General Dentistry, The Second Affiliated Hospital of Zhejiang University School of Medicine, Hangzhou, Zhejiang 310009, China

## Abstract

**Objective:**

This study aims to find the novel lncRNAs closely related to the progression of oral squamous cell carcinoma (OSCC) by comprehensively analyzing microarray.

**Methods:**

Chip dataset GSE84805 was downloaded from the Gene Expression Omnibus (GEO) database, lncRNA expression profiles of OSCC and paracancerous tissue were obtained, probes sequences reannotation was conducted, and differentially expressed lncRNAs (DELs) and differentially expressed genes (DEGs) were identified. Finally, these data were analyzed by constructing the lncRNA-function enrichment network.

**Results:**

We found that 465 lncRNAs are differentially expressed consisting of 193 upregulated lncRNAs and 272 downregulated lncRNAs. Meanwhile, 811 DEGs were identified with 498 upregulated genes and 313 downregulated genes. Analysis of the lncRNA-function enrichment network showed that these aberrant lncRNAs may be related to focal adhesion, inflammatory response pathway, cell cycle, matrix metalloproteinases, and other biological functions. Also, we found that some key lncRNAs such as LINC00152 and HOXA11-AS have been shown to play an important role in tumor proliferation and migration.

**Conclusion:**

The key lncRNAs may serve as potential molecular markers or therapeutic targets in OSCC formation and development. It can also help us to understand the molecular mechanism of occurrence and development in OSCC.

## 1. Introduction

Oral squamous cell carcinoma (OSCC), the 11th most prevalent cancer worldwide, accounts for more than 550,000 cases annually worldwide and is currently one of the leading causes of cancer-related death [1, 2]. Treatment of OSCC with surgery and adjuvant chemoradiation has improved the locoregional control rate of this disease [1, 3]. However, the control rate of distant metastasis and overall survival (OS) rates remain low [4, 5] and the mortality rates are still approximately fifty percent [5, 6]. The high mortality rate could be attributed to late diagnosis and lack of accurate biomarkers for predicting tumor progression and patient prognosis [7, 8]. Thus, a better understanding of the genetic and molecular disorders of the disease is the key to early diagnosis, appropriate treatment and improved prognosis of patients with OSCC.

Gene expression profiling provides a tool to search for biomarkers and explore the mechanism of development of OSCC [9, 10]. Potential candidate molecules can be found throughout the genome. Previous studies have focused on protein-coding genes, while recent studies have reported that long noncoding RNAs (200 nucleotides or longer) with a lack of coding potential, actually play critical biological roles in oral cancer [11]. For example, the expression of colon cancer-associated transcript 2 (CCAT2) was significantly higher in OSCC than that in adjacent tissues. Also, CCAT2 expression in low-differentiated OSCC was significantly higher than that in high-differentiated cancer. Therefore, upregulation of CCAT2 expression in tumor tissue might act as an oncogene and promote the development of OSCC [11–13]. Liu et al. found HOX transcript antisense intergenic RNA (HOTAIR) was highly expressed in OSCC, which facilitated the proliferation of OSCC Tca8113 cells and decreased their apoptosis. Thus, they identified HOTAIR as a qualified molecular marker for diagnosis and early warning of patients with OSCC [14–16].

Though a few lncRNAs have been functionally characterized, there are still a large number of functional transcripts which may have been unintentionally overlooked. In our study, we compare the expression of lncRNAs in paired tumor with normal tissues of OSCC based on the dataset GSE84805 deposited in the GEO (Gene Ontology Omnibus). We find some differentially expressed long noncoding RNAs (DELs) probably act as candidate biomarkers in OSCC. After lncRNA-function enrichment analysis, we point out the potential regulatory functions of lncRNAs. Our study provides new insights into the molecular discovery of OSCC that helps us understand the roles of lncRNAs in OSCC and further reveals the molecular mechanism of the development and progression of OSCC.

## 2. Methods

### 2.1. Microarray Data

The lncRNA and mRNA expression profiles of 6 OSCCs and 6 matched adjacent noncancerous tissues, deposited by Li and colleagues (accession number: GSE84805), were downloaded from GEO. The lncRNA and mRNA expression were detected by using an Arraystar human lncRNA microarray V3 (Arraystar Inc., Maryland, MD, USA). The raw txt data are downloaded, and the Quantile method is used to normalize the data.

### 2.2. Probes Sequences Reannotation

The probes sequences provided by the GEO platform (GPL16956) are aligned to long noncoding transcript sequences from the LNCipedia 4.0 database [17] and to the coding transcript sequences from the RefSeq database [18], respectively, using ncbi-blast-2.4.0+. The transcript sequences of 28980 lncRNA are matching with LNCipedia and the remaining unannotated 3855 lncRNAs are marked with seqname from GEO. The coding transcript sequences of 26022 mRNA are matching with RefSeq and the remaining unannotated 87 mRNAs are marked with seqname from GEO. These lncRNAs are then named after the HUGO symbol of the nearest protein-coding genes on the same strand using the LNCipedia name criterion.

### 2.3. Differential Expression Analysis

Raw signal intensity data are imported into BRB-ArrayTools version 4.5 (National Cancer Institute, http://linus.nci.nih.gov/BRB-ArrayTools.html) for preprocessing. In total, 32835 lnRNAs and 26109 genes are used for further analysis. We identify DELs and DEGs using a paired *T*-test with a nominal significance level for the local false discovery rate [19] being less than 0.05. Only lncRNAs and mRNAs with a fold change ≧ 2 are selected as DELs and DEGs.

### 2.4. Construction of lncRNA-Function Enrichment Network

The ENViz app is used in Cytoscape for lncRNA-function enrichment analysis [20]. ENViz performs joint enrichment analysis of gene expression and long noncoding RNA expression of sample matched datasets and available systematic annotations, such as pathway or gene ontology (GO) annotations in the following way. For each lncRNA, we rank elements of the gene expression data based on the correlation to the lncRNA expression across all samples, and compute statistical enrichment of annotation elements at the top of this ranked list based on the minimum hypergeometric statistics [21, 22]. Significant results are represented as an enrichment network, a bipartite graph with nodes corresponding to lncRNA and function annotation entries and edges corresponding to lncRNA-function annotation entry pairs with enrichment scores. We select an enrichment score threshold ≥4 as a cutoff to filter out the significant biological pathways using the WikiPathways database [23]. Furthermore, the enrichment score ≥5 and 8 are, respectively, selected as the threshold values of the significant molecular function and biological process based on gene ontology (GO) annotation. These edges of the enrichment network point to potential functionally relevant mechanisms. Cytoscape v3.4.0 [24]. is used to visualize the connected networks and enrichment information.

## 3. Results

### 3.1. Identification of DELs and DEGs in OSCC Patients

In order to investigate the differential expression of lncRNA and mRNA, we first compared the lncRNA or mRNA expression profiles of OSCC tissues and adjacent normal tissues using unsupervised hierarchical clustering (Figure 1(a), 1(b)). We found a total of 465 DELs with fold change ≧ 2 and FDR<0.05, including 193 upregulated lncRNAs and 272 downregulated lncRNAs (Table S1); Meanwhile, we identified 811 DEGs, including 498 upregulated mRNAs and 313 downregulated mRNAs with fold change ≧ 2 and FDR <0.05 (Table S2).

### 3.2. LncRNA-Function Enrichment Network

To exploring the critical biological roles of the lncRNAs in OSCC tumorigenesis and development, we integrated the lncRNAs and mRNA expression profiling data by using the power of enrichment statistics and knowledge of genomic annotation databases to assign relevant function annotations to gain better understating of the relationship between DELs and DEGs levels in the same sample. The lncRNA-pathways enrichment network showed that these DELs significantly enriched in some cancer-related pathways including focal adhesion, inflammatory response pathway, cell cycle, matrix metalloproteinases, and other biological functions (Figure 2). Interestingly, the adhesion pathway was the most relevant one (CumEnrichmentValue = 2454.11) and almost all (99.99%) the DELs were associated with focal adhesion pathways, and the most relevant lncRNAs were lnc-ZDHHC17-6 (*p*_*mHG*_=10^−9.49^), lnc-C7orf11-3 (*p*_*mHG*_=10^−8.63^), and lnc-MRPL39-2 (*p*_*mHG*_=10^−8.27^). There were 14 lncRNAs correlated along the inflammatory response pathway, out of which 79% (11/14) were upregulated and 21% (3/14) downregulated, and the most relevant lncRNAs were lnc-TMEM185B-2 (10^−4.97^), lnc-FAM8A1-2 (*p*_*mHG*_=10^−4.73^), and lnc-C18orf26-2 (*p*_*mHG*_=10^−4.56^). Here, 11 lncRNAs were related with cell cycle pathways, with 4 upregulated and 7 downregulated. Among that, lnc-CHAF1B-2 (*p*_*mHG*_=10^−5.94^), lnc-MED11-1 (*p*_*mHG*_=10^−5.95^), and lnc-TRIM29-2 (*p*_*mHG*_=10^−4.56^) were most relevant. Besides, there were upregulated lnc-C12orf39-1 (*p*_*mHG*_=10^−4.24^), downregulated lnc-KLHL31-2 (*p*_*mHG*_=10^−4.14^^4^), and lnc-AC136428.1.1–3 (*p*_*mHG*_=10^−4.90^) correlated to the matrix metalloproteinases.

We also performed joint enrichment analysis of lncRNA and the significant molecular function and biological process based on gene ontology (GO). Biological process analysis showed that 94% (436/465) DELs were enriched in the extracellular matrix organization and the extracellular structure organization (Figure 3). Among them, lnc-ZDHHC17-6 (*p*_*mHG*_=10^−16.52^), lnc-RP11-152F13.5.1–4 (*p*_*mHG*_=10^−16.35^), lnc-C18orf26-2 (*p*_*mHG*_=10^−15.94^), lnc-FCRL3-1 (*p*_*mHG*_=10^−15.83^), and lnc-SEC11A-6 (*p*_*mHG*_=10^−15.83^) were the most relative lncRNAs. Besides, molecular function analysis showed the most significant functional groups consisted of the lncRNAs involved in platelet-derived growth factor binding, metallopeptidase activity, and metalloendopeptidase activity (Figure 4).

## 4. Discussion

Previous studies of gene expression profiling have focused on the exploration of the functions of mRNAs, while we turn our attention to the long noncoding RNA which is no longer regarded as transcriptional noise and has recently been regarded as valuable transcripts in tumor progression and metastasis. For example, HOTAIR has been proven as a prognostic biomarker and therapeutic target in diverse human cancers, which promotes tumorigenesis and progression by the influence on reprogramming chromatin organization, histone demethylase, activating the promoter, and combination with microRNA to regulate downstream cancer-related molecules [25–27]. With the deepening of genome research, many new important molecules and mechanisms have been found. In particular, recent studies have shown that lncRNAs may play an important role in the occurrence and development of OSCC and may become a potential target for OSCC-targeted therapy. In OSCC, a number of lncRNAs, such as MALAT1 [28, 29], UCA1 [30, 31], FTH1P3 [32], PDIA3F, GTF2IRD2P1 [33], FOXC1, and FOXCUT [34] have been functionally identified, but compared to other cancers, the overall biological role and clinical significance of lncRNAs in OSCC remains largely unknown.

In our study, we identified 193 upregulated and 272 downregulated lncRNAs in patients with OSCC. Among those lncRNAs, FEZF1-AS1 [35], LUCAT1 [36], LINC00313 [37], and lnc-BCL2L11-3 [38] have been published their characteristics and functions in specific cancers. FEZF1-AS1 has been reported to facilitate cell proliferation and migration in colorectal carcinoma (CRC) and may play a role in the promotion of cancer by regulating the expression of sense-cognate gene FEZF1 mRNA and protein in CRC cells [35]. LUCAT1 in NSCLC (non-small cell lung cancer) tissues was proved obviously upregulated compared to normal tissues. LUCAT1 was confirmed to promote proliferation in vitro and in vivo and played a crucial role in G1 arrest as well [36]. LINC00313 was also proved upregulated in lung cancer tissues, compared with adjacent lung tissues and regarded as a poor prognosis biomarker for lung cancer [37]. Besides, lnc-BCL2L11-3 was found to be upregulated in the recurrent NPC tissues in comparison with the paired normal tissues, and the distinctive lncRNA identified in the recurrent NPC may reveal a distinctive development mechanism underlying tumor recurrence [38]. Those lncRNAs in supportive literature and our analysis have the same expression direction, which indicates that those lncRNAs may be potential biomarkers and therapeutic targets in OSCC, but we need larger samples for further validation.

In addition, we successfully constructed lncRNA-function enrichment network to analyze the functions of lncRNAs. Our analysis results show that DELs are mainly enriched in some pathways closely related to tumor progression, including focal adhesion, inflammatory response pathway, cell cycle, matrix metalloproteinases, and so on. Also, the adhesion pathway [39] turns out to be the most relevant pathway in our study. In the tumorigenesis of OSCC, focal adhesion, as one of the most important cellular transduction pathways, is located below the tight junction of the epithelial cells and helps cell-extracellular matrix (ECM) adhesion by resulting in changes into the actomyosin. In our lncRNA-function network, the focal adhesion pathway, as the center of the function network, connects 99.99% DELs and indirectly associates with other functional pathways, such as cell cycle and other relative pathways. It has been reported that among the lncRNAs, LINC00520, HOXA11-AS, and LINC00152 in other tumors associated with adhesion and cell cycle. Depletion of LINC00520 as reported results in decreased cell migration and loss of invasive structures in 3D may contribute to the molecular etiology of breast cancer [40]. HOXA11-AS highlighted alterations in cell proliferation and cell-cell adhesion pathways and enhanced cell proliferation, migration, and tumor invasion in vitro. Mechanistically, HOXA11-AS recruits the histone demethylase LSD1 or DNMT1 combining with E2H2 as a scaffold and promotes the progression and metastasis of gastric carcinoma [41, 42]. The cell cycle pathway is another important pathway in lncRNAs network. Wang et al. published that the HOXA11-AS transcript promoted cell proliferation via regulation of cell cycle progression in vitro [41, 42]. HOXA11-AS is upregulated in OSCC tissues in our analysis, corresponding with the results reported in other cancers [43]. Similarly, in various tumors, LINC00152 knockdown could inhibit cell proliferation and colony formation, trigger late apoptosis, and suppress cell migration and invasion [44–47].

In summary, some of lncRNAs associated with adhesion and cell cycle by network analysis have been supported in studies which proved that the methods of network-based function analysis by using lncRNA expression data is effective for understanding biomarker prediction and molecular mechanisms of OSCC. It may provide a new vision on therapeutic targets in OSCC by exploring the underlying mechanisms. Our research also has some limitations. First, we do not generate the microarray data by ourselves but took them from the GEO database. Second, there are few research studies on lncRNAs in OSCC, therefore lacking the verifications of other data sets or samples in our studies. Besides, we need to validate our results based on the experimental functional study.

## 5. Conclusion

In conclusion, this study demonstrated the effectiveness of network-based function analysis for understanding lncRNA biomarker prediction and molecular mechanisms of OSCC. These novel molecules for further investigation in development and progression may provide targets for future therapies in OSCC.

## Figures and Tables

**Figure 1:** Heat map of the 465 lncRNAs (a) and 811 genes (b) differentiating OSCC samples from noncancerous samples.

**Figure 2:** lncRNA-pathways enrichment network constructed using OSCC-related differentially expressed lncRNAs. Nodes are pathways (color-coded yellow or red by cumulative enrichment score) and lncRNAs (color-coded gray). Edges between pathway and lncRNA nodes are color-coded by direction of pathway-lncRNA correlation, red corresponds to positive, and blue corresponds to negative. Thickness of the edge is proportional to the enrichment score.

**Figure 3:** Enrichment network biological process based on gene ontology (GO). Nodes are biological process of GO term, colored on a yellow to red scale, according to the GO term cumulative enrichment value, and lncRNAs are colored gray, edges between GO term and lncRNA nodes are color-coded by direction of pathway-lncRNA correlation, red corresponds to positive and blue corresponds to negative. Thickness of the edge is proportional to the enrichment score.

**Figure 4:** Enrichment network molecular function based on gene ontology (GO). Nodes are molecular function of GO term, colored on a yellow to red scale, according to the GO term cumulative enrichment value and lncRNAs are colored gray, edges between GO term and lncRNA nodes are color-coded by direction of pathway-lncRNA correlation, red corresponds to positive and blue corresponds to negative. Thickness of the edge is proportional to the enrichment score.

## Data Availability

The datasets used and analyzed in this study are accessible upon request from the corresponding author.

## Abbreviations

OSCC: Oral squamous cell carcinoma
lncRNA: Long noncoding RNA
DELs: Differentially expressed lncRNAs
DEGs: Differentially expressed genes
GO: Gene ontology.

## Supplementary Materials

Supplementary Materials S1 table: differentially expressed lncRNAs. S2 table: differentially expressed genes.
